# Predicting Decreased Activities of Daily Living in Patients with Moyamoya Disease after Revascularization: Development and Assessment of a New Predictive Nomogram

This article has been retracted.

**DOI:** 10.1155/2021/6624245

**Published:** 2021-04-05

**Authors:** Yani Zhao, Dongliang Yang, Gang Li, Peng Zhao, Xiaorong Luan, Haiyan Li

**Affiliations:** ^1^Department of Neurosurgery, Qilu Hospital of Shandong University, Jinan 250012, China; ^2^Cangzhou Medical College, Cangzhou 061000, China; ^3^Department of Infection Management Office, Qilu Hospital of Shandong University, Jinan 250012, China

## Abstract

The aim of this study was to develop and validate a nomogram model to predict the risk of decreased activities of daily living (ADLs) in patients with moyamoya disease (MMD) following revascularization. The nomogram model was constructed based on data from 292 patients with MMD that were treated at Qilu Hospital of Shandong University from January 2018 to June 2019. The prediction model was assessed using a dataset of 119 patients with MMD collected from July 2019 to June 2020. Patients were evaluated with a general information questionnaire and the Mini Mental Status Examination, Hospital Anxiety and Depression Scale, Social Support Rating Scale, and ADL Scale. Multivariable logistic regression analysis was applied to build a prediction model incorporating the features selected in the least absolute shrinkage and selection operator regression model. Discrimination, calibration, and clinical usefulness of the prediction model were assessed using receiver operating characteristic (ROC) curves, calibration plots, and decision curve analysis. Predictors contained in the nomogram included gender, age, monthly income, hypertension, and cognitive function and depression scores. The areas under the ROC curves of the training and testing datasets were 0.938 and 0.853, respectively. The prediction model displayed good calibration, and the decision curve analysis showed that it had a wide range of clinical applications. This novel predictive could be conveniently used to predict the risk of the decreased living activity ability in patients with MMD.

## 1. Introduction

Moyamoya disease (MMD) is a chronic occlusive cerebrovascular disease characterized by progressive stenosis or occlusion of the bilateral internal carotid arteries, anterior cerebral arteries, and middle cerebral arteries; it often manifests as single or repeated attack of hemorrhagic or ischemic stroke [1, 2]. MMD has a relatively high incidence in East Asia [3]. Studies demonstrated that vascular reconstruction can effectively decrease the incidence of stroke [4, 5], but neurological dysfunction due to stroke, postoperative complications, and other reasons significantly influence patients' activities of daily living (ADLs) and even lead to disability [6]. This requires considerable social resources for rehabilitation and nursing, which places a heavy burden on both families and healthcare resources [7]. Therefore, it is important to predict and evaluate the postoperative ADLs of MMD patients.

ADLs are the daily activities that individuals perform to care for themselves and maintain their lives. The ability or inability to perform ADLs is an important functional measurement. It is also widely used to predict the prognosis and evaluate the self-care ability of stroke patients [8]. However, few studies have focused on the postoperative ADLs of patients with MMD. A model is needed to evaluate the survival status of patients after vascular reconstruction to determine which factors influence patient ADLs.

Nomograms are used to establish relevant prognostic models based on disease characteristics to predict patient outcomes. They have been widely used to predict survival [9]. However, few groups have used nomograms to predict the quality of life of patients after surgery for MMD.

In our study, we aimed to (i) explore the influencing factors and weights of ADL in patients with MMD after vascular reconstruction, (ii) develop and validate a prediction model for Chinese MMD patients, and (iii) use simple and effective nomograms to predict postoperative ADL status in MMD patients. This will enable us to prevent or reduce the occurrence of inability to perform ADL in MMD patients.

## 2. Materials and Methods

### 2.1. Patients

Study subjects were selected with a convenience sampling method. All the patients included in our study were treated in the Department of Neurosurgery of Qilu Hospital of Shandong University from January 2018 to June 2020. A face-to-face questionnaire survey was administered 3 months after surgery. The inclusion criteria were as follows: (i) age ≥ 18, (ii) diagnosed with MMD based on digital subtraction angiography, and (iii) vascular reconstruction with superficial temporal artery-middle cerebral artery bypass graft performed for the first time. Patients with other severe diseases, secondary vascular reconstruction, or severe cognitive dysfunction were excluded. The predictive model was constructed based on a training dataset including patients who met the inclusion criteria. The same inclusion criteria were used to select a testing dataset that included patients treated at Qilu Hospital of Shandong University between July 2019 and June 2020.

This study was approved by the Ethics Committee of Qilu Hospital of Shandong University (No. 2016.109), and informed consent was obtained from all patients.

### 2.2. Sample Size

The sample size was determined based on the principle that it should be 5-10 times the number of independent variables [10]. Our study included 21 variables, so the sample size should be at least 210. Based on the estimation that ~20% of patients would reject the questionnaire, we determined the sample size should be at least 252.

### 2.3. Research Methods

#### 2.3.1. General Data Questionnaire

We designed the general data questionnaire based on the information and characteristics of MMD. It included gender, age, monthly income, hypertension, diabetes, heart disease, and many other factors. The diagnosis of complications was confirmed by two doctors according to clinical diagnostic criteria.

#### 2.3.2. ADL Scale

ADLs were evaluated with the ADL scale, which consists of 14 items including physical activity ability (including 6 items like eating and dressing) and instrumental daily activity ability (including 8 items such as taking buses and shopping). Each item was scored as 1-4 points. A score ≥ 14 was considered to indicate a decline of ADLs. The Cronbach's alpha of this scale was 0.940.

#### 2.3.3. Mini Mental Status Examination (MMSE)

The MMSE was used to test cognitive function. It has 30 items that queries abilities in 5 dimensions (orientation, attention, computing power, recall ability, and language ability). Each item is scored as 0 or 1 point, with a total score of 0 to 30 points. The Cronbach's alpha of this scale was 0.743.

#### 2.3.4. Hospital Anxiety and Depression Scale (HADS)

The HADS is a reliable tool for evaluating anxiety and depression. It is divided into two subscales (anxiety and depression), with seven items in each. The Cronbach's alpha of the anxiety and depression subscales were 0.817 and 0.832, respectively.

#### 2.3.5. Social Support Rating Scale (SSRS)

This scale has good reliability and validity in evaluating the degree of social support in patients with cerebrovascular disease. There are 3 dimensions (subjective support, objective support, and utilization of support) and 10 items. The Cronbach's alpha of the scale was 0.812.

### 2.4. Statistical Analysis

Statistical analysis was performed using R software (Version 3.4.4). Normally distributed data are presented as the means and standard deviations ($\bar{x}\pm s$), and quantitative data are expressed as frequency and percentage (%). The least absolute shrinkage and selection operator (LASSO) method was used to select optimal predictive features among risk factors. Features with nonzero coefficients in the LASSO regression model were selected; then multivariable logistic regression analysis was used to build a prediction model by incorporating the selected features. All potential predictors were applied to develop a model to predict decreased ADL risk. The discrimination, calibration, and clinical usefulness of the predicting model were assessed using receiver operative characteristic (ROC) curves, calibration plots, and decision curve analysis. The specific research process is shown in Figure 1.

## 3. Results

### 3.1. Patient Characteristics

A total of 411 patients with MMD were included in our study, with 292 patients in the training dataset and 119 patients in the testing dataset. The male : female ratio was balanced, and the patients ranged in age from 23 to 66, with a mean age of 50.11 ± 10.04 years old. Nearly 60 percent of patients had decreased ADL postoperatively. The general characteristics of the patients in the training and testing sets are shown in Table 1.

### 3.2. Identifying Independent Predictors

Seven potential predictors were identified with LASSO regression, including gender, age, family per capita monthly income, hypertension, cognitive function, depression, and social support scores (Figure 2). These variables were incorporated into multivariate logistic regression, which revealed six independent predictors. As shown in Table 2, females, patients with hypertension, older age, and higher depression scores increased the risk of ADL decline. Conversely, patients with higher income and good cognitive function were at the lower risk of decreased ADL.

### 3.3. Development and Evaluation of the Nomogram Prediction Model

According to the multivariate logistic regression analysis, six independent predictors (gender, age, monthly income, hypertension, cognitive function, and depression scores) were combined to develop the nomogram risk prediction model (Figure 3). The assignment and scores of each predictor are shown in Table 3. In this study, the calibration curves (Figure 4) of the ADL risk prediction model for MMD patients were generated in both the training and testing datasets. The results showed good consistency and a high degree of calibration, indicating that the prediction model was more accurate. Then the ROC curves of the prediction model in the training and testing data sets were analyzed to evaluate the model's diagnostic effect (Figure 5). The areas under the ROC curves in both groups were >0.8, suggesting that this model could predict postoperative ADLs in MMD patients. The decision curve analysis indicated that the prediction model had a wide range of applications (Figure 6). Collectively, the findings show that the nomograph prediction model constructed with the above six indicators had an accurate predictive value for ADLs in MMD patients.

## 4. Discussion

ADLs are an important indicator to evaluate the recovery of MMD patients who experienced a stroke. It is crucial to identify high-risk subjects in advance and provide timely interventions, therefore improving their quality of life. We developed and validated a prediction model for MMD patients by evaluating ADLs. Predictors contained in the nomogram included gender, age, monthly income, hypertension status, and cognitive function and depression scores; it can help clinicians determine the high-risk population and provide a foundation for sound medical treatment. We also validated our nomogram using ROC curves, calibration plots, and decision curve analysis.

Our study showed that ~60% of MMD patients with revascularization had decreased ADLs, which was in accordance with a previous study [11]. Because decreased ADLs significantly influence patient quality of life, it is important to clarify which factors are associated with the ADLs of MMD patients who underwent vascular reconstruction. However, few studies have focused on the postoperative prognosis of MMD patients. We evaluated the ADLs of MMD patients following revascularization and identified the factors that affected patient ADLs by focusing on general demographics, clinical data, psychology, and sociology. The variables of this model are easy to obtain and integrate multiple predictive variables into the line diagram, which is intuitive and convenient for calculation.

The six predictive factors included in the nomogram deserve more attention from medical workers, especially the cognitive function and depression scores. We found that MMD patients with lower cognitive function were more likely to have decreased ADLs after surgery. Some researchers posited that cognitive dysfunction would influence ADLs in MMD patients [12]. Another study showed that cognitive impairment seriously affected patient quality of life [13]. A possible reason is that the typical pathological changes of MMD include stenosis or occlusion of critical arteries resulted in long-term chronic cerebral ischemia and stroke, therefore influencing cognitive function. Other studies reported that vascular reconstruction did not improve cognitive function [14, 15], and the patients usually had impairments in executive function, concentration, memory, computing power, and logistical ability, all of which decrease independent living abilities.

Depression is a common complication of cerebrovascular disease, especially stroke. As a unique chronic progressive cerebrovascular disease, MMD is likely to induce depression [16]. We found that depression was an important factor that contributed to decreased ADL, which was in accordance with Ezema et al.'s study [17]. Since depressed patients experience negative emotions and a lack of confidence, motivation, and enthusiasm to participate in daily activities, ADL recovery is changing. Moreover, depression is likely to contribute to cognitive impairment, which further influences ADL recovery [16, 17].

Previous studies based on normal populations demonstrated that patients with hypertension were more likely to have decreased ADLs [18, 19]. We also found that hypertension was an independent risk factor for decreased ADLs in MMD patients. A reasonable explanation may be that hypertensive patients face the risk of functional decline, and there are more complications leading to the decline of ADL function [18]. Furthermore, it was reported that hypertension could increase the risks of ADL decline, postoperative cerebral infarction, and complications, which can result in muscle strength decline, aphasia, and other neurological issues.

General demographic data such as gender, age, and income were identified as key predictive factors for ADL. We found that females were more likely to have decreased ADL after surgery for MMD. Several previous studies also reported that female patients had worse prognoses and lower ADLs than male patients [20–22]. This may be due to the fact that female patients have weaker constitutions and are less able to withstand emergent events. MMD is more likely to be diagnosed in children and young adults, and the risk of postoperative ADL decline increases with age [23]. Conversely, higher family income was associated with a reduced likelihood of decreased ADL. This result was not completely in accordance with previous research, and the reason may be that most patients in our study were low-income residents from rural areas.

In view of the high rate of acute ADL decline in MMD patients and the current lack of predictive tools, clinicians can use this model to predict patient ADL status. The possible clinical application is to strengthen cognitive training, pay more attention to psychological factors, encourage patients to actively accept treatment, and address depression symptoms. Moreover, it is also important to control blood pressure in patients with MMD to maintain the cerebral perfusion. Furthermore, women, older patients, and those with low income should be considered high-risk populations and closely followed.

Our results should be considered in the context limitations. The data were collected at a single research center, although they were relatively systematic and complete. And the prediction model was validated using patient data from the same research center, which may partly reduce its generalizability.

## 5. Conclusion

We developed a novel prediction model to determine the risk of decreased ADLs in MMD patients following revascularization. This nomogram incorporates gender, age, monthly income, hypertension status, and cognitive function and depression scores and can be conveniently used to predict the risk of the decreased ADLs in patients with MMD. Based on this nomogram, interventions and treatments could be employed to prevent decreased ADLs and improve patient quality of life.

## Figures and Tables

**Figure 1:** Research process flow chart.

**Figure 2:** Variable selection using the LASSO regression model. (a) The selection of the best parameter in the LASSO model (lambda) uses a 10-fold cross-validation approach. (b) Seven variables with coefficients not equal to zero were selected through LASSO regression.

**Figure 3:** Nomogram for predicting declined ADLs.

**Figure 4:** Establishment and validation of the prediction model. (a) The prediction model was calibrated in the training dataset. (b) The prediction model in the validation set of the calibration diagram. Note: the *x*-axis represents the prediction risk of ADL function decline, the *y*-axis represents the actual risk of ADL function decline, the diagonal dashed line represents the ideal prediction effect of the theoretical model, and the solid line represents the performance of the nomogram. A closer diagonal dashed line indicates a stronger prediction effect.

**Figure 5:** ROC curves of the predictive model. (a) Training dataset model. (b) Testing dataset model.

**Figure 6:** Decision curve of the prediction model.

**Table 1:** General characteristics of the training and testing sets.

Variables	Training set (*n* = 292)		Testing set (*n* = 119)	
	Number of cases/($\bar{x}\pm s$)	%	Number of cases	%
Gender				
Male	146	50	60	50.4
Female	146	50	59	49.6
Age				
≤44	87	29.8	35	29.4
45-59	140	47.9	59	49.6
≥60	65	22.3	25	21.0
Level of education				
Never attended school	36	12.3	13	10.9
Primary or junior high school	172	58.9	68	57.1
Senior high school and above	84	28.8	38	32.0
Marital status				
Married	283	96.9	113	95.0
Unmarried/divorced/widowed	9	3.1	6	5.0
Residence				
City	93	31.8	36	30.3
Village	114	39.0	48	40.3
County/town	85	29.1	35	29.4
Profession				
Physical labor	121	41.4	40	33.6
Professional worker	90	30.8	47	39.5
Retired/unemployed	19	6.5	12	10.1
Other career	62	21.2	20	16.8
Payment				
Worker healthcare	136	46.6	54	45.4
Resident healthcare	147	50.3	49	41.2
Other	9	3.1	16	13.4
Household per capita monthly income				
≤1000 RMB	112	38.4	45	37.8
1001-3000 RMB	80	27.4	30	25.2
>3000 RMB	100	34.2	44	37.0
Lesion type				
Cerebral hemorrhage	124	42.5	52	43.7
Cerebral ischemia	168	57.5	67	56.3
Cerebral infarction				
Yes	88	30.1	34	28.6
Diabetes				
Yes	34	11.6	21	17.6
Hypertension				
Yes	94	32.2	41	34.5
Heart disease				
Yes	13	4.5	12	10.1
Time between disease onset and surgery				
≤6 weeks	74	25.3	31	26.1
6-12 weeks	115	39.4	49	41.2
>12 weeks	103	35.3	39	32.8
Operation side				
Right	123	42.1	52	43.7
Postoperative complications				
Yes	24	8.2	14	11.8
Regular exercise				
No	150	51.4	52	43.7
Cognitive function score	23.75 ± 5.00		23.98 ± 4.53	
Anxiety score	5.53 ± 3.34		5.10 ± 3.01	
Depression scores	6.78 ± 3.87		6.42 ± 3.46	
Social support score	37.58 ± 6.48		36.31 ± 6.95	
Decreased ability in daily life	178	61.0	67	56.3

**Table 2:** Multivariate logistic regression results regarding decreased ADLs in patients with MMD.

Variable	Odds ratio (95% confidence interval)	*P*
Female gender	2.24 (1.06, 4.84)	0.037
Age	2.19 (1.30, 3.77)	0.004
Family per capita monthly income	0.44 (0.26, 0.72)	0.002
Hypertension	4.04 (1.74, 9.87)	0.001
Cognitive function score	0.61 (0.50, 0.73)	<0.001
Depression score	1.30 (1.12, 1.51)	0.001

**Table 3:** Values assigned to each variable in the nomogram model.

Variable	Assignment	Score/risk factor
Gender	1 = male	0
	2 = female	8
Age	0 ≤ 44	0
	1 = 45-59	8
	2 ≥ 60	16
Household per capita monthly income	0 ≤ 1000 RMB	17
	1 = 1001-3000 RMB	8
	2 ≥ 3000 RMB	0
Hypertension	1 = no	0
	2 = yes	14
Cognitive function score	10	100
	20	50
	30	0
Depression score	0	0
	10	27
	20	54
Total score	35	Risk of ADL decline = 0.1
	57	Risk of ADL decline = 0.5
	66	Risk of ADL decline = 0.7

## Data Availability

Source data are available from the corresponding author upon reasonable request.
